# A Meta-Analysis on the Effectiveness of Video Laryngoscopy versus Laryngoscopy for Emergency Orotracheal Intubation

**DOI:** 10.1155/2022/1474298

**Published:** 2022-01-07

**Authors:** Xiaotong Ba

**Affiliations:** Department of Emergency Internal Medicine, Daxing District People's Hospital (Capital Medical University Daxing Teaching Hospital), Beijing, China

## Abstract

**Background:**

Video laryngoscopy has been associated with some orotracheal intubations and enhances the glottic view at time of laryngoscopy and the success rate of the intubation in patients from the emergency department and the intensive care unit. In usual cases, direct laryngoscopy is performed among the patients from the emergency department or the intensive care unit. In this systematic review and meta-analysis, we draw the comparison between the video laryngoscopy and direct laryngoscopy for the emergency orotracheal intubation.

**Objective:**

The objective of the study was to identify the clinical efficacy of video laryngoscopy versus laryngoscopy for emergency orotracheal intubation.

**Materials and Methods:**

MEDLINE, CENTRAL, EMBASE, and Web of Science databases were analyzed from 2003 to 2020. Keywords used for searching the studies were “laryngoscopy,” “video laryngoscopy,” “direct laryngoscopy,” “emergency department,” “intensive care unit,” “orotracheal,” “video laryngoscope,” “glidescope,” “airway scope,” “airway,” “Macintosh laryngoscopy,” “airway management,” “tracheal intubation,” “orotracheal intubation,” and “intubation.”

**Results:**

The first-pass intubation success rates in the intensive care unit were low in video laryngoscopy with 95% CI 1.21 (1.13–1.30) and heterogeneity *I*2 = 78% favoring direct laryngoscopy nonsignificantly with low heterogeneity. Odds ratio for airway trauma or dental damage was 0.67, 95% CI (0.18–2.54), reported higher in video laryngoscopy. Complications with oesophageal laryngoscopy were higher in video laryngoscopy with risk ratio 0.16, 95% CI (0.09–0.29), odds ratio 0.88, 95% CI (0.65–1.18) for sever hypoxemia, risk ratio 1.53, 95% CI (1.02–2.28) for cardiovascular collapse, risk ratio with 95% CI 1.11 (0.59–2.07) for aspiration complications, and odds ratio 1.32, 95% CI (0.95, 1.85) for Inexperienced medical staff handling laryngoscopy.

**Conclusion:**

No significant efficiency was noticed in using video laryngoscopy when compared with direct laryngoscopy with the available data. The data reported in studies are not enough for efficient clinical analysis of the benefits of using video laryngoscopy over direct laryngoscopy. Thus, information such as length of stay, mortality, sever complications, and length of hospital stay must be reported.

## 1. Introduction

The video laryngoscopy (VL) is recommended in the guidelines of airway administration to encourage the tracheal intubation [1]. The hypothetical advantages of the video laryngoscopy are engaging in the administration of the patients who necessitate emergency orotracheal intubation. Although, there do exist conditions where the direct laryngoscopy turns beneficial over the video laryngoscopy (for an instance when functioned by skilful clinicians). Moreover, the advanced glottis visualization with the video laryngoscopy might not be necessarily able to translate into an excessive success for the first-pass intubation because the tracheal intubation turns out to be arduous under the indirect sight.

The tracheal intubation is an important process for lifesaving carried out in the emergency department or the intensive care unit (ICU) for the patients who are suffering with respiratory disorders or a lower airway protection [2].

In any urgent situation, the airway administration can be challenging because of the heart failure physiology, deficit supply of tools and qualified staffs, disconnected state, parallel performance of the cardiopulmonary resuscitation (CPR) or other related medical course of action, inappropriate approach to the patient's head, and multiple anatomic characteristics of tough airways [3].

It has been investigated that the rate of failure of the urgent tracheal intubations in the emergency department or intensive care unit is remarkably more than that of the tracheal intubations performed in the operating room [4]. The video laryngoscopy for the endotracheal intubation might issue a fine laryngeal visualization [5], but how much of it is rendered into a clinical interest such as reduced intubation duration, inflated success rate of intubation, or few hurdles is questionable.

A review study from Cochrane identified that the video laryngoscopy is linked with considerably small failure rate and its outcome dimensions expand in the patients with expected tough airway. Video laryngoscopy is a novel tool which consists of a small camera over the tip of the blade for indirect visualization of the glottis.

Because of the verified benefits of a fast-learning curve, an enhanced laryngeal visualization, and an expanded rate of success, video laryngoscopy has been extensively utilized for tracheal intubation during the extremity and grave conditions [6–10].

There have been multiple meta-analyses drawing the comparison of video laryngoscopy versus the laryngoscopy for emergency orotracheal intubation in the patients admitted in the emergency department and the intensive care unit and yield varied results [11, 12]. There is still lack of clarity whether the utilization of video laryngoscopy can diminish the detrimental events linked with tracheal intubations in the patients from the emergency department and intensive care unit (Figure 1).

## 2. Materials and Methods

Articles that were rejected as per their exclusion criteria: no outcome, insufficient patient data, nonclinical studies, review papers, studies that lacked location and pediatric population, abstracts, and letters or editorials = 117.

### 2.1. Search Strategy

This systematic review and meta-analysis developed the directions of the Preferred Reporting Items for Systematic Reviews and Meta-Analysis (PRISMA) assertion for performing and documenting outcomes. A systematic literature search was conducted referring to MEDLINE, Cochrane Central Register of Controlled Trials (CENTRAL), EMBASE, and Web of Science in the duration of 2003 to 2020.

The studies documented in the English language were considered for analysis, and we also considered published review articles as well as editorials as the additional records identifiable for our study.

### 2.2. Eligibility Criteria and Inclusion Factors

The studies that were published as the prospective randomized control trials which documented the comparisons of video laryngoscopy with direct laryngoscopy among the patients of the emergency department and the intensive care unit. The observational studies comparing the video laryngoscopy and direct laryngoscopy demonstrating the harmful cases of tracheal intubations in the patients of the intensive care unit were also included.

The following keywords were used to search the database: “laryngoscopy,” “video laryngoscopy,” “direct laryngoscopy,” “emergency department,” “intensive care unit,” “orotracheal,” “video laryngoscope,” “glidescope,” “airway scope,” “airway,” “Macintosh laryngoscopy,” “airway management,” “tracheal intubation,” “orotracheal intubation,” and “intubation.”

### 2.3. Exclusion Criteria

The exclusion criteria were as follows: the studies where video laryngoscopy or direct laryngoscopy was utilized as a saving device; the studies that were prehospital studies or simulated studies; the patient data which had information about doubtful laryngeal trauma or an excess of maxillofacial wound with a need of urgent surgical airway; and the studies that had duplicate data.

## 3. Results

Table 1 summarizes the characteristics of the selected studies on the basis of given parameters of country of study, study type, hospital setting, intubation type, video laryngoscopy type, medical experts, and age of patients in both video laryngoscopy and direct laryngoscopy.

Table 2 summarizes the comparative analysis of video laryngoscopy and direct laryngoscopy over the first-pass intubation success rate in the intensive care unit.

Figure 2 represents the risk ratio determination for video laryngoscopy vs. the direct laryngoscopy for six studies [7, 13–17], for 1312 and 737 cases of VL and DL, respectively, wherein 95% CI is 1.21 (1.13–1.30) and heterogeneity I^2^ = 78% (CI, confidence interval; DL, direct laryngoscopy; and VL, video laryngoscopy).

Figure 3represents the scattered plot for the first-pass intubation for the success ratio in the intensive care unit patients using the funnel plot analysis.

Table 3 represents the video laryngoscopy and direct laryngoscopy for the four studies [7, 14–16] with respect to the airway trauma or the dental damage.

In Figure 4, the four studies [7, 14–16] were analyzed for the odds ratio where 95% CI is 0.67 (0.18–2.54) and heterogeneity *I*^2^ = 0%; the video laryngoscopy and direct laryngoscopy were examined with respect to the airway trauma or the dental damage during the procedure for 1382 and 737 events of VL and DL, respectively (CI, confidence interval; DL, direct laryngoscopy; and VL, video laryngoscopy).

Figure 5 represents the scattered plot of the airway trauma or the dental damage procedure using the funnel plot analysis for all cases from the given studies.

Table 4 represents the comparative analysis of methods of video laryngoscopy vs. the standard direct laryngoscopy for five studies [7, 14–17] for cases of oesophageal laryngoscopy.

In Figure 6, the forest plot analysis over the complex cases of oesophageal laryngoscopy measured the risk ratio by comparing the video laryngoscopy and the direct laryngoscopy techniques, where we observed 95% CI 0.16 (0.09–0.29) and heterogeneity *I*^2^ = 62%; CI, confidence interval; DL, direct laryngoscopy; and VL, video laryngoscopy.

Table 5 represents the comparison of techniques of video laryngoscopy vs. the standard technique (direct laryngoscopy) where different cases were reported in the studies conducted in [7, 13, 15–17]. The comparison of the both the techniques represents cases facing sever hypoxemia as the complication of intubation.

In Figure 7, the forest plot analysis of the incidents with severe hypoxemia with respect to the complication of intubation showcases the process results for methods video laryngoscopy vs. the direct laryngoscopy, wherein 95% CI observed with odds ratio was 0.88 (0.65–1.18) and the heterogeneity measures to be *I*^2^ = 44% (Figure 7); CI, confidence interval; DL, direct laryngoscopy; and VL, video laryngoscopy.

Table 6 represents the different cases observed in the abovementioned six studies [7, 13–17], wherein these cases were observed experiencing cardiovascular collapse as the complication of intubation. The comparison of cases under video laryngoscopy vs. the direct, i.e., the standard, laryngoscopy was measured as per the cases.

Figure 8 represents the forest plot analysis of the incidents that experience the cardiovascular collapse as the complication of intubation. Here, these six studies define the risk ratio comparing the video laryngoscopy vs. the standard laryngoscopy, wherein the observed 95% CI = 1.53 (1.02–2.28) and heterogeneity *I*^2^ = 0%; CI, confidence interval; DL, direct laryngoscopy; and VL, video laryngoscopy.

Figure 9 demonstrates the scattered plot of the effect which showcases the estimated analysis of the test cases with the cardiovascular collapse as the incident of complication of intubation.

Table 7 represents the comparative analysis of the abovementioned six studies [7, 13–15, 17], wherein the two techniques video laryngoscopy vs. direct laryngoscopy are differentiated with respect to the complicated cases of procedural complexities in aspiration.

In Figure 10, the forest plot analysis for the abovementioned six studies demonstrates the risk ratio for the comparative analysis of video laryngoscopy and the direct laryngoscopy over the complicated cases of the procedural complexities in aspiration, where the 95% CI = 1.11 (0.59–2.07) and heterogeneity *I*^2^ = 0%; CI, confidence interval; DL, direct laryngoscopy; and VL, video laryngoscopy.

Figure 11 demonstrates the scattered plot of the effect which showcases the estimated analysis of the test cases on complicated cases of procedural complications in aspiration.

Table 8 represents the comparative analysis of the abovementioned three studies [13, 16, 17], wherein the two techniques video laryngoscopy vs. direct laryngoscopy are differentiated with respect to the inexperienced medical staff assistance while handling laryngoscopy.

In Figure 12, the forest plot analysis for the abovementioned three studies demonstrates the risk ratio for the comparative analysis of video laryngoscopy and the direct laryngoscopy over the complicated cases of the procedural complexities in aspiration, where the 95% CI = 1.32 (0.95–1.85) and heterogeneity *I*^2^ = 81%, and the total events were reported as 225 and 208 for video laryngoscopy and direct laryngoscopy, respectively (CI, confidence interval; DL, direct laryngoscopy; and VL, video laryngoscopy).

In Figure 13, the success rate of two studies [13, 16] represented the 95% CI for 1.01 [0.70, 1.48] odds ratio for a total of 184 events for each video laryngoscopy and direct laryngoscopy techniques for the overall effect; *Z* = 0.08 for *P* = 0.94, on the basis of Macintosh-type laryngoscopy blades in both VL and DL (CI, confidence interval; DL, direct laryngoscopy; and VL, video laryngoscopy).

## 4. Discussion

The first-pass intubation success rates in the intensive care unit using video and direct laryngoscopy was analyzed where the success rates of video laryngoscopy were low with 95% CI 1.21 (1.13–1.30) and heterogeneity *I*^2^ = 78% favoring direct laryngoscopy nonsignificantly with low heterogeneity; details of the case are shown in Table 2, a forest plot of analysis is shown in Figure 2, and a funnel plot is shown in Figure 3. Hence, direct laryngoscopy gave good results.

Airway trauma or dental damage caused due to laryngoscopy procedures were analyzed. Odd ratio for 95% CI were 0.67 (0.18–2.54) with no heterogeneity. Nonsignificant results were obtained with higher incidences of airway trauma or dental damage in video laryngoscopy, thereby favoring direct laryngoscopy. The details of the study are shown in Table 3, a forest plot of analysis is shown in Figure 4, and a funnel plot is shown in Figure 5. Direct laryngoscopy gave better outcomes as they reported lesser damage.

Complications with oesophageal laryngoscopy were higher in video laryngoscopy in comparison to direct laryngoscopy with risk ratio 0.16, 95% CI (0.09–0.29), and low heterogeneity 62%. The number of complicated cases was reported as shown in Table 4, a forest plot of the analysis is shown in Figure 6, and a funnel plot is shown in Figure 14. Complications were higher in video laryngoscopy; hence, it is not a preferable method.

Cases facing severe hypoxemia as a complication of intubation were reported higher in video laryngoscopy when compared with direct laryngoscopy with odds ratio 0.88, 95% CI (0.65–1.18), and very low heterogeneity *I*^2^ = 44%. The cases reported are shown in Table 5 with forest plot analysis in Figure 7 and a funnel plot in Figure 15.

Cases experiencing cardiovascular collapse as complications of intubation were higher in direct laryngoscopy when compared with video laryngoscopy as shown in Table 6 with forest plot analysis in Figure 8 and a funnel plot in Figure 9. Risk ratio was 1.53, 95% CI (1.02–2.28), with no heterogeneity *I*^2^ = 0%; hence, the results are not significant.

Complicated cases of procedural complications in aspiration were analyzed where direct laryngoscopy reported higher risk ratio with 95% CI 1.11 (0.59–2.07). Results were not significant with no heterogeneity *I*^2^ = 0%. Data are shown in Table 7, forest plot analysis is shown in Figure 10, and a funnel plot is shown in Figure 11. Inexperienced medical staff handling laryngoscopy favored direct laryngoscopy nonsignificantly with odds ratio 1.32 95% CI (0.95, 1.85), and a forest plot is shown in Figure 12. Success rates on the basis of Macintosh-type laryngoscope blades in laryngoscopy were analyzed by a forest plot as in Figure 13 with odds ratio 1.01 (0.70,1.48).

## 5. Conclusions

In this meta-analysis, we have analyzed the efficacy and complications suffered in cases with video laryngoscopy when compared with direct laryngoscopy. The first-pass intubation success rates in the intensive care unit were better in direct laryngoscopy though nonsignificant. The first attempt rates were analyzed, and multiple attempts increase the risk, thus making it complicated. Usually a highly experienced anesthesiologist shows better superiority unless a case of difficult airway is experienced, thereby leading to more success rates [18].

There are plenty other factors which may further elaborate the difference in effectiveness between video or direct laryngoscopy. As patients who are critically ill are subjected to poor oxygen reserved, they are more subjected to hypoxia making the operators opt for direct laryngoscopy or mask oxygenation. Secretions, fluids, and blood in the airway can block the airway from getting clouded, thus impairing visualization in the larynx. Increased term of intubation is a major cause for increasing mortality in patients who are undergoing intubation prior to hospitalization. Mostly direct laryngoscopy is easily assessable to operators in prehospitalization cases.

In this systematic review, no significant improvements were noted in video laryngoscopy when compared with direct laryngoscopy. The first-pass intubation success rates in the intensive care unit were better in direct laryngoscopy. Airway trauma or dental damage, oesophageal laryngoscopy, and severe hypoxemia are other complications in intubation reported higher in video laryngoscopy. Thus, intubation outcomes may be worsened by using video laryngoscopy.

Hence, more studies need to be performed for determination of benefits of video laryngoscopy for emergency or critical care in patients regardless of any operator's experience. Furthermore, the impacts such as length of stay, mortality, sever complications, and length of hospital stay must be reported for an efficient and clinical analysis of determining the benefits of using video laryngoscopy over direct laryngoscopy.

## Figures and Tables

**Figure 1:** PRISMA study over the study methods.

**Figure 2:** First-pass intubation success rates in the intensive care unit forest plot.

**Figure 3:** First-pass intubation success rates in the intensive care unit funnel plot.

**Figure 4:** Forest plot for analysis of airway trauma or dental damage during the procedure.

**Figure 5:** Funnel plot for analysis of airway trauma or dental damage during the procedure.

**Figure 6:** Forest plot on complicated cases with oesophageal laryngoscopy.

**Figure 7:** Forest plot of cases facing severe hypoxemia as a complication of intubation.

**Figure 8:** Forest plot of cases experiencing cardiovascular collapse as complications of intubation.

**Figure 9:** Funnel plot on cases experiencing cardiovascular collapse as complications of intubation.

**Figure 10:** Forest plot on complicated cases of procedural complications in aspiration.

**Figure 11:** Funnel plot on complicated cases of procedural complications in aspiration.

**Figure 12:** Forest plot of inexperienced medical staff handling laryngoscopy.

**Figure 13:** Success rates on the basis of Macintosh-type laryngoscope blades in video and direct laryngoscopy.

**Figure 14:** Funnel plot on complicated cases with oesophageal laryngoscopy. CI, confidence interval; DL, direct laryngoscopy; and VL, video laryngoscopy.

**Figure 15:** Funnel plot of cases facing severe hypoxemia as a complication of intubation.

**Table 1:** Characteristics of studies.

Studies	Characteristics					
	[7]	[13]	[14]	[15]	[16]	[17]
**Country of study**	USA	USA	France	USA	France	Israel

**Study type**	Propensity matched analysis	Randomized clinical trial	Observational	Observational	Randomized clinical trial	Randomized clinical trial

**Hospital setting**	Intensive care unit	Intensive care unit	Intensive care unit	Intensive care unit	Intensive care unit	Intensive care unit

**Intubation type**	Emergency intubations	Emergency intubations	Emergency intubations	Emergency intubations	Emergency intubations	Emergency intubations

**Video laryngoscopy type**	Multiple	McGRATH/GlideScope/Olympus	McGRATHMAC	GlideScope	McGRATHMAC	GlideScope

**Medical experts**	6 doctors (postgraduate)	Pulmonary experts and critical care supervised by physicians	ICU physicians and anesthetists	Pulmonary critical care experts and intensive care unit	ICU physicians	Pulmonary and critical care experts

**Age, yrs (VL)**	59 (49–69)	59 (49–68)	63 (55–70)	66 ± 16.96	62.7 (15.3)	65.4

**Age, yrs (DL)**	60 (53–73)	60 (51–67)	59 (49–69)	69 ± 16.88	62.8 (16.3)	69.6

**Total number**	809	150	210	392	371	153

**Table 2:** Comparison of first-pass intubation success rates in the intensive care unit.

Studies	Video laryngoscopy		Direct (standard) laryngoscopy	
	Cases	Total	Cases	Total
[7]	541	673	89	136
[14]	55	70	96	140
[13]	58	74	54	76
[15]	199	252	75	140
[16]	126	186	130	185
[17]	41	57	24	60

**Table 3:** Airway trauma or dental damage during the procedure.

Studies	Video laryngoscopy		Direct (standard) laryngoscopy	
	Cases	Total	Cases	Total
[7]	4	673	0	136
[14]	0	70	0	140
[15]	2	252	2	140
[16]	0	387	1	322

**Table 4:** Complicated cases with oesophageal laryngoscopy.

Studies	Video laryngoscopy		Direct (standard) laryngoscopy	
	Cases	Total	Cases	Total
[7]	13	673	7	136
[13]	1	74	4	76
[15]	1	252	27	140
[16]	3	186	6	185
[17]	0	57	4	60

**Table 5:** Number of cases facing severe hypoxemia as a complication of intubation.

Studies	Video laryngoscopy		Direct (standard) laryngoscopy	
	Cases	Total	Cases	Total
[7]	123	673	35	136
[13]	14	74	16	76
[15]	30	252	9	140
[16]	20	186	20	185
[17]	2	57	5	60

**Table 6:** Cases experiencing cardiovascular collapse as complications of intubation.

Studies	Video laryngoscopy		Direct (standard) laryngoscopy	
	Cases	Total	Cases	Total
[7]	54	673	6	136
[13]	8	74	7	76
[14]	6	70	8	140
[15]	16	252	4	140
[16]	8	186	4	185
[17]	6	57	8	60

**Table 7:** Complicated cases of procedural complications in aspiration.

Studies	Video laryngoscopy		Direct (standard) laryngoscopy	
	Cases	Total	Cases	Total
[7]	14	673	3	136
[13]	1	74	1	76
[14]	0	70	2	140
[15]	5	252	2	140
[16]	4	186	4	185
[17]	6	57	4	60

**Table 8:** Inexperienced medical staff handling laryngoscopy.

Studies	Video laryngoscopy		Direct (standard) laryngoscopy	
	Cases	Total	Cases	Total
[13]	58	74	54	76
[16]	126	186	130	185
[17]	41	57	24	60

## Data Availability

The data used to support the findings of this study are available from the corresponding author upon request.
